RETRACTED

# Appraising and reacting to voluntary green behavior at work: The effects of green motive attribution

**DOI:** 10.3389/fpsyg.2022.1010588

**Published:** 2022-09-26

**Authors:** Xue Zhang, Zhongqiu Li, Huilai Zhang, Qiwen Zhang

**Affiliations:** ^1^College of Philosophy, Law and Political Science, Shanghai Normal University, Shanghai, China; ^2^College of Economics and Management, Northeast Agricultural University, Harbin, China; ^3^School of Marxism, Harbin University of Science and Technology, Harbin, China

**Keywords:** green behavior, attribution theory, warmth, green advocacy, work psychology

## Abstract

Starting from the perspective of social perception of voluntary employee green behavior (VEGB) and studies on the attribution of VEGB, we explore the phenomenon that employees can show different perceptions and behavioral responses to VEGB according to their attribution to VEGB. We served to examine the hypotheses. The results of a two-wave study show that when employees believe VEGB is motivated by instrumental concerns, VEGB is more likely to evoke a low level of warmth and competence, which produces less green advocacy. However, if employees believe VEGB is motivated by moral reasons, VEGB is more likely to prompt more warmth and competence perceptions and elicit greener advocacy from employees. In addition, theoretical and practical contributions are discussed.

## Introduction

Recently, companies have become increasingly committed to protecting the environment and the proper management of natural resources to develop their economic, social, and environmental assets and realize their goal of ecological sustainability (Buysse and Verbeke, 2003; Sihvonen and Partanen, 2017; Wang et al., 2018a). Businesses and individuals recognize the seriousness of the ecological problem and demand the introduction of sustainable operations. In particular, the pioneering role of humans in environmental protection has attracted many organizations (Starik and Marcus, 2000; Yan et al., 2021). Employees who care about the environment tend to engage in many eco-friendly behaviors at work, such as paper recycling, printing on both sides of the page, and conserving water and electricity (Safari et al., 2018; Zhang et al., 2021). Voluntary employee green behavior (VEGB) is recognized as an effective path to organizational environmental sustainability that has attracted the attention of scholars in recent years (Galpin and Whittington, 2012; Norton et al., 2015; Yue et al., 2020). As a type of environmentally friendly behavior, VEGB refers to employee acts that support environmental sustainability within the company but are not under the control of a formal environmental management policy or system (Ones and Dilchert, 2012; Norton et al., 2015). It can also be seen as an employee acting outside of their scope of work by taking the initiative to engage, going above and beyond what is expected of them by the organization, and fostering sustainability in the workplace environment (Tian et al., 2020; Chen et al., 2021). Given its contribution to an organization’s sustainable development, most researchers have attempted to understand the antecedents of VEGB, such as human resource practice (Haddock-Millar et al., 2016), organizational strategy (Norton et al., 2017), and leadership (Robertson and Barling, 2013; Khan et al., 2019; Tian and Robertson, 2019). While research exists on the outcomes of VEGB, little is known about how coworkers respond to VEGB. This represents an essential gap in the literature on why employees respond differently and what factors influence their different reactions. In this study, we try to shed light on the impact of VEGB by combining the ideas of warmth and competence perception, which are essential to comprehending how coworkers perceive VEGB. Previous studies have demonstrated that individuals evaluate others based on their warmth and competence (Fiske et al., 2007; Cuddy et al., 2008). In this study, we suggest that warmth and competence are the underlying mechanisms that explain VEGB.

RETRACTED

We offer an alternative perspective and argue that not all coworkers believe VEGB is a good activity. Our arguments align with research that demonstrated that sometimes employees regard pro-social behavior negatively (Maon et al., 2019). Moreover, few studies have shown that coworkers’ perceptions can be biased (Mitchell et al., 2015; Causadias et al., 2018). This study has demonstrated that the manner in which coworkers react depends on how they perceive VEGB’s motivation. To clarify coworkers’ responses to VEGB, we build on attribution theory. According to attribution theory, individuals make inferences about others, and that one’s perceptions of motivation can influence their subsequent behavior (Martinko et al., 2011). According to attribution, coworkers analyze employees’ motives for getting involved in VEGB. Previous research has identified two categories of motives that influence coworkers’ attitudes and behavior: pro-environment motives and self-interest motives (Chang et al., 2019). In this research, we propose that perceived motives of green initiatives will moderate the relationship between VEGB and perception (perceived warmth and competence). To improve the managerial implications of our findings, we included coworker green advocacy as an outcome variable in the model. Coworker green advocacy is the degree to which coworkers publicly discuss environmental sustainability, exchange pertinent information, and express their varied viewpoints to persuade others to engage in environmentally friendly behavior (Kim et al., 2017; Shujie et al., 2022). It reflects the eco-friendly ambiance characterized by social interactions, distinct from the personal initiative in the pursuit of work (Frese and Fay, 2001). We contend that employees’ VEGB may incite coworker green advocacy. Likewise, when coworkers observe an employee’s VEGB, coworkers may be inclined to endorse that behavior to demonstrate their shared concern and build a closer bond with the employee, leading to coworker green advocacy as a result. This research aims to investigate the relationship between VEGB and coworker green advocacy (Figure 1).

RETRACTED

**FIGURE 1:** Research model.

Our findings make three contributions to the literature. First, our research extends the knowledge by explaining why VEGB motives different coworkers’ reactions. Although much of the work on VEGB has examined its effect from the actors’ perspectives, we suggest that not all coworkers react to VEGB similarly because not all coworkers hold the same beliefs about the employees engaging in VEGB. Second, we extend the knowledge of coworkers’ reactions to VEGB. Scholars repeatedly address calls to examine the outcomes of VEGB (Ren et al., 2018). We address this call by showing the link between VEGB and coworker green advocacy. We offer a crucial clarification of social perception by showing how coworkers’ reactions depend on their beliefs of VEGB actors. Therefore, we refine social perception to consider necessary boundary conditions about the impact of coworkers’ reactions to VEGB. Third, we introduce a psychological mechanism (i.e., perceived warmth and competence) to explain the impact of VEGB on coworker green advocacy. The findings of this study will help the organization to understand the influence of perceived warmth and competence of VEGB performers, as well as the attributed motives of green initiatives, on coworker green advocacy. We clarify the underlying mechanisms and boundary conditions through which VEGB translated into coworker green advocacy. Our findings inform organizations that investing in VEGB is worthwhile, as it improves coworker green advocacy.

## Literature review and hypotheses

### Voluntary employee green behavior and coworker perception

Organizations heavily rely on the actions of their employees to accomplish environmental sustainability. Previous researchers stressed the need to encourage environmentally responsible behavior in the workplace (Bissing-Olson et al., 2013). VEGB is one of the tactics used by organizations to achieve sustainability goals and improve environmental performance. VEGB evolves from employee green behavior (EGB), which refers to environmentally beneficial behavior that protects and even benefits the environment in the workplace (Ones and Dilchert, 2013). EGB is pro-social and can be segregated into two dimensions: one is the required EGB; that is, employees engage in environmentally friendly conduct following corporate policies and standards. The other is VEGB; employee-initiated green behavior goes above and beyond what is expected of the organization and is not constrained by its formal guidelines.

RETRACTED

Given that individuals have varying degrees of control over how to engage in these activities at work, required EGB and VEGB may have different antecedents, even though both are deemed crucial to achieving the organization’s green goals (Dumont et al., 2017). However, according to Ones and Dilchert (2012), most green workplace behaviors are voluntary. VEGB is more esoteric and can consist of recommendations as simple as turning off lights at the end of the day to improve the organization’s environmental performance (Paillé and Boiral, 2013). According to Norton et al. (2015), VEGB should incorporate practices like shutting off the electricity while leaving the office (i.e., conserving energy), recycling reusable materials at work (i.e., recycling), and revising papers electronically rather than printing them out (i.e., avoiding waste) (Tian et al., 2020). Therefore, we focus on VEGB, a type of pro-environmental behavior that helps mitigate the detrimental effects of human activity (Ones and Dilchert, 2012).

In this study, we suggest that VEGB might be seen as warm and competent. Before examining the association between VEGB and coworker perception, the perceived warmth and competence mentioned above need to be first defined. The literature on social perception often involves two fundamental dimensions: warmth and competence perception (Fiske et al., 2002; Abele and Wojciszke, 2014). Perceived warmth is typically believed to include traits of morality and sociability, such as kindness, friendliness, and good nature. In contrast, perceived competence is frequently seen to possess qualities of skills, such as ability, efficiency, and intelligence (Fiske et al., 2007). Warmth is essential for achieving non-specific, fundamental, and enduring goals like integrity, well-being, or social acceptance (Montoya and Horton, 2014). In general, warmth perception refers to being warm, compassionate, understanding, and showing concern for other people and society (Abele et al., 2008). VEGB actors can be perceived as environmentally conscious (Millar and Baloglu, 2011). Perceived competence influences the assessment of the ability of others to implement their motives effectively (Cuddy et al., 2011). Competent individuals strive to be independent and in control of their environment, are high performers, and tend to lead and dominate others. Hence, it may be said that warm people are more socially focused, whereas competent people are more individualistic and task-focused.

RETRACTED

### Moderating effect of perceived motives of green initiatives

Voluntary employee green behavior, which can positively influence organizational sustainability, is particularly likely to trigger an evaluation process regarding how coworkers’ interpretations of VEGB qualify what social perception might be evoked by VEGB. As mentioned, the social psychology perspective on appraisal contends that competence and warmth are crucial to comprehending how perceivers voluntarily interpret information about others (Schilpzand et al., 2022). The assessment focuses on developing the underlying motivations for VEGB. Although much of the VEGB research has been conducted with the implicit assumption that VEGB has pro-environmental intentions (Lalot et al., 2019) and is therefore evaluated as such, the construct of VEGB is not defined in terms of how third parties might perceive these motives. Thus, it is crucial to consider the likelihood that different coworkers may have different perspectives on the underlying motivation for VEGB. The belief that VEGB can be self-serving is evident in recent theorizing by environmental psychology scholars (Wang et al., 2018b). Indeed, the literature on green behavior has recently shifted from models that focus on principled moral motives to models that consider instrumental motives of organizational actors across various fields, such as management studies (Xu et al., 2021). For example, Paulraj and Chen (2007) proposed that there may be three types of causal attributions that drive firms to pursue green activities: instrumental, relational, and moral motives. This study claims that there are two motives, instrumental and moral, that might encourage employees to embrace VEGB practices. Instrumental attribution refers to individuals who perceive VEGB to be driven by self-interest. In contrast, moral attribution refers to individuals who perceive VEGB to be motivated by a desire to concern with ethical standards and moral principles. Coworkers may make assumptions about employees’ purpose for engaging in VEGB when evaluating their VEGB. Therefore, coworkers may perceive and respond to VEGB differently depending on how much employees maintain instrumental or moral attributions for VEGB.

RETRACTED

When coworkers perceive VEGB as motivated by a desire to be concerned with ethical standards and moral principles, we hypothesized that warmth and competence perception are likely outcomes. A moral attribution for VEGB suggests that employee integrity can transcend laws and regulations to promote sustainable development. Employees bring their moral values to the workplace beyond economic self-interest. Some employees choose responsible activities like VEGB practices because it is the right thing to do (Cameron et al., 2004). They consider it their ethical obligation to improve the environment and society. Previous studies assume that individuals have moral obligations to behave responsibly. More particularly, many employees adhere to a set of values that view sustainability initiatives as a moral obligation. Thus, moral motives morally inspired employees to practice VEGB because of their intrinsic beliefs and sincere concern for the environment, but not due to social pressure. According to previous research, if someone is seen as having good intentions, they are likely to be stereotyped as warm and competent (Fiske et al., 2002). As noted above, some coworkers may view VEGB as stemming from a desire to protect the environment. Therefore, when coworkers interpret VEGB as driven by moral motives, we theorize that a high level of warmth and competence perception are the likely appraisal reaction to VEGB.

However, it is possible that not every coworker will believe employees’ VEGB stems from a desire for moral motivation. Business ethics scholars argue that in addition to moral motivations, employees’ VEGB is heavily influenced by instrumental motivations (Aguilera et al., 2007). Specifically, employees participate in VEGB out of self-interest or based on reciprocity (e.g., to attain a positive reputation). Accordingly, studies have demonstrated that perceived instrumental motives influence individuals’ responses (Barone et al., 2000). For instance, Chernev and Blair (2015) have shown that the beneficial effects of social goodwill are mitigated by perceived self-interest. Previous studies have asserted that employees will engage in green initiatives, such as VEGB, when these practices align with instrumental interests of protecting an individual’s impression so that employees can raise their negative impression (Aguilera et al., 2007). Previous studies have shown that when environmental initiatives like the VEGB are aligned with instrumental interests, employees will not support them, increasing their negative opinions of the actor. Instrumental motives are a type of consequentialism in which accountability is established by considering the effects of decisions (Anscombe, 1958). Conversely, in a VEGB setting, coworker-attributed instrumental intentions result in more unfavorable views than moral motives (Luo and Bhattacharya, 2006). In other words, coworkers are more likely to perceive a low level of warmth and competence for VEGB when attributing instrumental motives (Berens et al., 2007).

RETRACTED

In summary, we suggest that whether VEGB evokes a high level of warmth and competence perception depends on whether coworkers make an instrumental or a moral attribution. Specifically, the more a coworker attributes VEGB to an instrumental motive, the lower the perception of warmth and competence. The more a coworker attributes VEGB to a moral motive, the greater the perception of warmth and competence. Therefore, we hypothesize:

**Hypothesis 1a:** The relationship between VEGB and perceived warmth is moderated by coworker-attributed instrumental motives, such that the relationship is more positive when coworker-attributed instrumental motives are lower than when the motives are higher.

**Hypothesis 1b:** The relationship between VEGB and perceived competence is moderated by coworker-attributed instrumental motives, such that the relationship is more positive when coworker-attributed instrumental motives are lower than when the motives are higher.

**Hypothesis 2a:** The relationship between VEGB and perceived warmth is moderated by coworker-attributed moral motives, such that the relationship is more positive when coworker-attributed moral motives are higher than when the motives are lower.

**Hypothesis 2b:** The relationship between VEGB and perceived competence is moderated by coworker-attributed moral motives, such that the relationship is more positive when coworker-attributed moral motives are higher than when the motives are lower.

### Coworker green advocacy as outcome

As indicated above, VEGB interacts with individual differences in coworkers’ attribution to produce differential social perceptions. We now go into more detail about how these social perceptions, perceived warmth and competence, result in later behavioral responses. Many sociological and social-psychological studies have found that such perceptions of warmth and competence lead to different behavioral outcomes (Kim et al., 2020; Schilpzand et al., 2022). However, only a few studies on organizational behavior have looked at the role that social perceptions play in the context of green conduct. Researchers need to investigate how coworkers’ perceived warmth and competence could yield differing subsequent behavioral responses, such as coworker green advocacy, which represents pro-environment behavior that benefits sustainability (Hu et al., 2022). Coworker green advocacy states the extent to which coworkers amenably converse environmental challenges and potential solutions, exchange green knowledge, bring ecological issues to the attention of others, and persuade others to take an interest in ecological benefit behavior (Crucke et al., 2022). Coworkers’ values, convictions, and actions will exhibit a zone of flexibility influenced by the VEGB context. Specifically, employees provide green clues through their external activities and statements that could aid others to gather and interpreting information to regulate their behavior (Groth et al., 2002). Coworkers frequently rely on these green cues and match their behavior to these advocacies. Therefore, coworker green advocacy is shaped by the social perception of the employees and is varied according to the different ascribed motives of the VEGB. VEGB reinforces the significance of coworker green advocacy for organizations by fostering an eco-friendly workplace culture, enhancing environmental performance, and eventually attaining sustainable organizational development (Shujie et al., 2022). Although it benefits the environment and the company, little research has been done on the antecedents of their coworkers’ green advocacy (Wu and Cheng, 2017). In this study, we propose that perceived warmth and competence play a crucial role in employee behavioral response. In particular, we attempt to investigate whether the effect of perceived warmth and competence on coworker green advocacy is the same when coworkers attribute different motives for VEGB.

RETRACTED

When coworkers attribute the VEGB to moral motives, they are more likely to perceive warmth and competence, which elicit more coworker green advocacy. When coworkers observe employees exhibiting VEGB and attribute moral motives, higher warmth and competence are signaled, in that the VEGB actors can take care of both themselves and the environment (Becker-Olsen et al., 2006). Coworkers feel that VEGB performers genuinely care about the environment and consider that preserving the environment is the “right thing to do.” When VEGB is desired and appreciated by coworkers, they may be inspired to engage in pro-environmental behaviors (Ones and Dilchert, 2012). Coworkers are more likely to adopt virtues from actors (e.g., a sense of environmental responsibility) and engage in green advocacy, which will increase and reinforce the social support for the VEGB actors. For instance, if a coworker notices employees utilizing spreads for printouts, shutting off the lights when they leave the office, and making coffee with their own cups rather than disposable ones, they might start doing the same. Therefore, coworkers are more likely to adopt green advocacy practices in the workplace if they believe employees are environmentally responsible and act following VEGB that is morally motivated.

RETRACTED

In contrast, when coworkers attribute VEGB practices were motivated by an instrumental intention, they are less likely to have positive warmth and competence perception, which elicits less coworker green advocacy. Self-serving motivations affect evaluations of an employee’s VEGB efforts (Vlachos et al., 2009) and coworkers’ willingness to support green initiatives. Coworkers tend to assume that VEGB actors are trying to manipulate the impressions of others and develop negative attitudes toward them as a result. According to Grant and Mayer’s (2009) research, people may think less favorably of disingenuous, unreliable, and calculating employees. Thus, when employees see VEGB, they may be less inclined to endorse that behavior as an expression of shared concern, making them less likely to engage with green interests. Therefore, we expect coworkers who perceive actors as low in warmth and competence are less likely to take green advocacy actions. We offer the following integrative hypotheses:

**Hypothesis 3a:** VEGB is related to decreased coworker green advocacy through perceived warmth when coworker-attributed instrumental motives are lower than when the motives are higher.

**Hypothesis 3b:** VEGB is related to decreased coworker green advocacy through perceived competence when coworker-attributed instrumental motives are lower than when the motives are higher.

**Hypothesis 4a:** VEGB is related to increased coworker green advocacy through perceived warmth when coworker-attributed moral motives are higher than when the motives are lower.

**Hypothesis 4b:** VEGB is related to increased coworker green advocacy through perceived competence when coworker-attributed moral motives are higher than when the motives are lower.

## Method

### Sample and data collection

We recruited 300 participants with the assistance of managers of an industrial and commercial bureau in a southern province of China. Data were collected randomly from individuals working in full-time positions in various industries, including finance, education, and information technology. In our research, we used a critical incident methodology. It is difficult to effectively examine respondents’ reactions to specific events in a general survey. Previous literature recommends using critical incident techniques to focus the study on specific actors’ behavior and respondent reactions to a particular event (Hershcovis and Reich, 2013). This method is valid and useful for assessing peoples’ perceptions and responses (Mitchell et al., 2015). In the first survey, individuals were required to be working full-time, have witnessed employee VEGB within the past 12 months, and provide the initial of the employee in that situation. Afterward, participants were required to respond to a demographic survey online (such as age, gender, education, and tenure), their attributed instrumental motives, moral motives, perceived warmth, and perceived competence of this employee. One week later, we contacted the participants and asked them to complete a survey about green advocacy.

RETRACTED

A total of 246 participants took the Time 1 survey (82% response rate). Participants who said they had not directly observed the VEGB of employees were excluded from the data and the analysis. The final sample consists of 232 respondents invited to the Time 2 survey. Of these, 190 participants completed the Time 2 survey (81.90% response rate). At the same time, participants who miss completed an attention check item were removed from the analysis, leaving a final sample of 182 employees (78.45% response rate). The average age of the participants was 31.69 years, and 45.05% were male. Their employment lasted an average of 8.1 years.

### Measurement

Following the translation–back translation procedure (Brislin, 1970), we created Chinese versions of the measures. All survey responses used in our study range from 1 = “strongly disagree” to 5 = “strongly agree.”

Voluntary employee green behavior: The employees completed a six-item VEGB measure adapted from Robertson and Barling (2013). The sample items were “He/she prints double-sided whenever possible” and “He/she turns lights off when not in use.” “He/she put recyclable material in the recycling bins.” The Cronbach’s alpha coefficient was 0.70.

Coworker perceived warmth: We adopted three items from Fiske et al.’s (2002) scale. The sample items were “He/she is warm,” “He/she is good-natured,” and “He/she is friendly.” The Cronbach’s alpha coefficient was 0.73.

Coworker perceived competence: We adopted three items from Fiske et al.’s (2002) scale. The sample items were “He/she is competent,” “He/she is intelligent,” and “He/she is competitive.” The Cronbach’s alpha coefficient was 0.78.

Coworker-attributed instrumental motives: We adopted three questions developed by Paulraj et al.’s (2017) scale. The sample items were as follows: “He/she engages in green activities to enhance his or her image,” “He/she engages in green activities to build up favors for a later exchange,” and “He/she engages in green activities to create a good impression.” The Cronbach’s alpha coefficient was 0.80.

Coworker-attributed moral motives: We adopted four questions developed by Paulraj et al.’s (2017) scale. The sample items were as follows: “He/she participates in eco-friendly activities out of a sense of environmental responsibility,” “He/she practices green habits because of a sincere concern for the environment,” “He/she participates in green initiatives because senior managers view environmental responsiveness as an essential component of corporate strategy,” and “He/she practices green behavior because it is the right thing to do.” The Cronbach’s alpha coefficient was 0.70.

RETRACTED

Coworker green advocacy: We adopted three questions developed by Kim et al.’s (2017) scale. The sample items were as follows: “I made an effort to get others to recycle and repurpose office materials at work,” “I collaborate with my colleagues to create a more ecologically friendly workplace,” and “I share knowledge, information, and suggestions with my colleagues on how to prevent pollution at work.” The Cronbach’s alpha coefficient was 0.71.

Control variables: Previous research has shown that demographic characteristics may influence employees’ cognitions and attitudes at work (Ng and Feldman, 2012). Thus, we controlled for employees’ age, gender (0 = female, 1 = male), education, and tenure.

## Results

Table 1 shows the mean values, standard deviations, and correlation among the variables. We first used Mplus 8.3 software to conduct confirmatory factor analysis to examine the dimensionality of the six constructs representing VEGB, coworker-attributed instrumental motives, coworker-attributed moral motives, coworker perceived warmth, coworker perceived competence, and coworker green advocacy. The results revealed that the six-factor model fits the data well (ratio χ^2^/df = 1.46, CFI = 0.94, TLI = 0.92, RMSEA = 0.05, SRMR = 0.06) and better than all the other alternative models (see Table 2).

**TABLE 1:** Results of confirmatory factor analysis.

Model	χ^2^	df	χ^2^/df	CFI	TLI	RMSEA	SRMR
6-factor^a^	199.81	137	1.46	0.94	0.92	0.05	0.06
5-factor^b^	314.93	142	2.22	0.83	0.79	0.08	0.08
4-factor^c^	354.05	146	2.43	0.79	0.76	0.09	0.08
3-factor^d^	511.26	149	3.43	0.64	0.58	0.12	0.11
2-factor^e^	567.12	151	3.76	0.58	0.53	0.12	0.11
1-factor^f^	596.77	152	3.93	0.56	0.50	0.13	0.11

*n* = 182.

^a^All items were influenced by their own factors, respectively.

^b^Items for coworker perceived warmth and coworker perceived competence were influenced by the same factor, and items for other variables were influenced by their own factors respectively.

^c^Items for coworker green advocacy and VEGB were influenced by the same factor, coworker perceived warmth and coworker perceived competence were influenced by the same factor, and items for other variables were influenced by their own factors, respectively.

^d^Items for coworker green advocacy and VEGB were influenced by the same factor, coworker perceived warmth and coworker perceived competence were influenced by the same factor, and items for other variables were influenced by the same factor.

^e^Items for coworker green advocacy, VEGB, coworker perceived warmth, and coworker perceived competence were influenced by the same factor, and items for other variables were influenced by the same factor.

^f^There is only one factor influencing all variables.

*p < 0.05, **p < 0.01(two-tailed).

RETRACTED

**TABLE 2:** Descriptive statistics, correlations, and square roots of AVE.

Variables	*M*	*SD*	1	2	3	4	5	6	7	8	9
1. Gender	1.56	0.50	1								
2. Age	31.69	7.49	−0.19*	1							
3. Education	2.91	0.54	0.04	−0.18*	1						
4. Work tenure	8.10	7.00	−0.19**	0.96**	−0.23**	1					
5. VEGB	4.32	0.36	−0.08	0.18*	0.03	0.14	1				
6. Coworker attributed instrumental motives	3.59	0.93	−0.03	−0.01	0.07	−0.05	0.14	1			
7. Coworker attributed moral motives	4.41	0.39	−0.05	0.13	−0.02	0.12	0.52**	−0.03	1		
8. Coworker perceived warmth	4.42	0.49	−0.08	0.09	0.11	0.08	0.22**	−0.12	0.28**	1	
9. Coworker perceived competence	4.37	0.45	−0.11	0.11	−0.02	0.10	0.39**	−0.06	0.35**	0.22**	1
10. Coworker green advocacy	4.19	0.53	−0.06	0.19**	0.01	0.15*	0.49**	0.03	0.39**	0.40**	0.42**

*n* = 182. Gender: 0 = Male; 1 = Female.

*p < 0.05, **p < 0.01.

Table 3 presents a summary of the linear regression results. We conducted the regression with coworkers’ perceived warmth as the dependent variable. The results revealed that the interactive effect of VEGB and coworker-attributed instrumental motives on coworker perceived warmth was significant (*b* = −0.34, SE = 0.08, *p* < 0.01, Δ*R*^2^ = 0.12). The interactive effect of VEGB and coworker-attributed moral motives on coworker perceived warmth was also significant (*b* = 0.16, SE = 0.06, *p* < 0.01, Δ*R*^2^ = 0.07). Simple slopes analysis demonstrated that, when coworker-attributed instrumental motives were high, the relationship between VEGB and coworker perceived warmth was negative and significant (*t* = −1.98, *p* < 0.10). When coworker-attributed instrumental motives were low, the relationship between VEGB and coworker perceived warmth was positive and significant (*t* = 4.81, *p* < 0.01) (see Figure 2). When coworker-attributed moral motives were high, the relationship between VEGB and coworker perceived warmth was positive and significant (*t* = 7.16, *p* < 0.01). When coworker-attributed moral motives were low, the relationship between VEGB and coworker perceived warmth was not significant (*t* = 0, n.s.) (see Figure 3).

**TABLE 3:** Summary of multiple regression analysis results.

Variable	Coworker perceived warmth						Coworker perceived competence						Coworker green advocacy							
	Model 1		Model 2		Model 3		Model 4		Model 5		Model 6		Model 7		Model 8		Model 9		Model 10	
	*B*	*SE*	*B*	*SE*	*B*	*SE*	*B*	*SE*	*B*	*SE*	*B*	*SE*	*B*	*SE*	*B*	*SE*	*B*	*SE*	*B*	*SE*
Gender	−0.06	0.07	−0.02	0.08	−0.04	0.07	−0.07	0.07	−0.06	0.07	−0.06	0.07	−0.00	0.07	0.03	0.06	0.03	0.06	0.01	0.06
Age	−0.08	0.26	0.10	0.25	−0.02	0.25	0.01	0.25	0.09	0.25	0.06	0.25	0.40	0.24	0.42	0.21	0.41	0.22	0.38	0.21
Education	0.11	0.08	0.12	0.07	0.11	0.07	−0.02	0.07	−0.01	0.07	−0.02	0.07	−0.01	0.07	−0.03	0.06	−0.04	0.06	−0.03	0.06
Work tenure	0.15	0.27	−0.01	0.25	0.08	0.26	0.02	0.25	−0.06	0.25	−0.03	0.25	−0.30	0.24	−0.35	0.22	−0.34	0.22	−0.32	0.21
VEGB	0.20**	0.08	0.09	0.08	0.16	0.09	0.38**	0.07	0.35**	0.08	0.33	0.09	0.46**	0.07	0.32**	0.07	0.32**	0.07	0.18	0.07
Coworker perceived warmth															0.28**	0.06	0.29**	0.07	0.32**	0.06
Coworker perceived competence															0.22**	0.07	0.23**	0.07	0.25**	0.06
Coworker attributed instrumental motives			−0.12	0.07					−0.10	0.07							0.02	0.06		
Coworker attributed moral motives					0.25**	0.08					0.21**	0.08							0.04	0.07
VEGB * Coworker attributed instrumental motives			−0.34**	0.08					−0.10	0.08							0.02	0.07		
VEGB * Coworker attributed moral motives					0.16**	0.06					0.11*	0.06							−0.20**	0.05
*R* ^2^	0.07*		0.19**		0.14**		0.16**		0.18**		0.21**		0.26**		0.39**		0.40**		0.45**	
Δ*R*^2^			0.12**		0.07**				0.02		0.05**				0.13**		0.01		0.06**	

*n* = 182. Gender: 0 = Male; 1 = Female.

*p < 0.05, **p < 0.01.

RETRACTED

**FIGURE 2:** The interactive effect of VEGB coworker-attributed instrumental motives on perceived warmth.

**FIGURE 3:** The interactive effect of VEGB coworker-attributed moral motives on perceived warmth.

Then, we conducted the regression with coworker perceived competence as the dependent variable. The results revealed that the interactive effect of VEGB and coworker-attributed instrumental motives on coworker perceived competence was not significant (*b* = −0.10, SE = 0.08, n.s., Δ*R*^2^ = 0.02). The interactive effect of VEGB and coworker-attributed moral motives on coworker perceived competence was significant (*b* = 0.11, SE = 0.06, *p* < 0.01, Δ*R*^2^ = 0.05). Simple slopes analysis demonstrated that, when coworker-attributed instrumental motives were high, the relationship between VEGB and coworker perceived competence was significant (*t* = 5.03, *p* < 0.01). When coworker-attributed instrumental motives were low, the link between VEGB and coworker perceived competence was positive and significant (*t* = 1.98, *p* < 0.05) (see Figure 4). When coworker-attributed moral motives were high, the relationship between VEGB and coworker perceived competence was positive and significant (*t* = 13.91, *p* < 0.01). When coworker-attributed moral motives were low, the relationship between VEGB and coworker perceived competence was not significant (*t* = 1.93, n.s.) (see Figure 5). We obtained the same findings when the control variables were removed from the model. Thus, Hypotheses 1a, 2a, and 2b were proven, and Hypothesis 1b was not confirmed.

RETRACTED

**FIGURE 4:** The interactive effect of VEGB coworker-attributed instrumental motives on perceived competence.

**FIGURE 5:** The interactive effect of VEGB coworker-attributed moral motives on perceived competence.

We predicted that coworker perceived warmth and competence would mediate the interaction effect between VEGB and coworker-attributed motives (instrumental motives vs. moral motives) on coworker green advocacy. We tested for moderated mediation using Model 7 of the PROCESS macro (Hayes et al., 2017) to generate bootstrap confidence intervals (see Table 4). When coworker-attributed instrumental motives were high, the indirect effect of VEGB on coworker green advocacy through coworker perceived warmth was significant (indirect effect = −0.10, SE = 0.06, 95% CI [−0.24, −0.01]). When coworker-attributed instrumental motives were low (1 SD below the mean), the indirect effect of VEGB on coworker green advocacy through coworker perceived warmth was also significant (indirect effect = 0.17, SE = 0.06, 95% CI [0.07, 0.30]). The CI of index of moderated mediation was not included as zero (*b* = −0.15, SE = 0.06, 95% CI [−0.27, −0.05]). When coworker-attributed moral motives were high, the indirect effect of VEGB on coworker green advocacy through coworker perceived warmth was significant (indirect effect = 0.13, SE = 0.07, 95% CI [0.02, 0.27]). When coworker-attributed moral motives were low, the indirect effect of VEGB on coworker green advocacy through coworker perceived warmth was not significant (indirect effect = −0.00, SE = 0.05, 95% CI [−0.11, 0.08]). The CI of index of moderated mediation was not included as zero (*b* = 0.17, SE = 0.07, 95% CI [0.04, 0.33]). Thus, Hypotheses 3a and 4a were proven.

**TABLE 4:** Conditional indirect effects.

Mediator	Moderator	Level	Effect	SE	95% CI
Coworker perceived warmth	Coworker attributed instrumental motives	Low	0.17	0.06	[0.07, 0.30]
		High	−0.10	0.06	[−0.24, 0.01]
		Index of moderated mediation	−0.15	0.06	[−0.27, −0.05]
	Coworker attributed moral motives	Low	−0.00	0.05	[−0.11, 0.08]
		High	0.13	0.07	[0.02, 0.27]
		Index of moderated mediation	0.17	0.07	[0.04, 0.33]
Coworker perceived competence	Coworker attributed instrumental motives	Low	0.15	0.05	[0.06, 0.26]
		High	0.08	0.05	[0.00, 0.18]
		Index of moderated mediation	−0.04	0.03	[−0.01, 0.02]
	Coworker attributed moral motives	Low	0.07	0.03	[0.02, 0.14]
		High	0.14	0.05	[0.05, 0.25]
		Index of moderated mediation	0.09	0.04	[0.03, 0.18]

*n* = 182.

RETRACTED

When coworker-attributed instrumental motives were high, the indirect effect of VEGB on coworker green advocacy through coworker perceived competence was significant (indirect effect = 0.08, SE = 0.07, 95% CI [0.02, 0.27]). When coworker-attributed instrumental motives were low, the indirect effect of VEGB on coworker green advocacy through coworker perceived competence was significant (indirect effect = 0.15, SE = 0.05, 95% CI [0.06, 0.26]). The CI of index of moderated mediation was included as zero (*b* = −0.04, SE = 0.03, 95% CI [−0.01, 0.02]). When coworker-attributed moral motives were high, the indirect effect of VEGB on coworker green advocacy through coworker perceived competence was significant (indirect effect = 0.14, SE = 0.05, 95% CI [0.05, 0.25]). When coworker-attributed moral motives were low, the indirect effect of VEGB on coworker green advocacy through coworker perceived competence was not significant (indirect effect = 0.07, SE = 0.03, 95% CI [0.02, 0.14]). The CI of index of moderated mediation was not included as zero (*b* = 0.09, SE = 0.04, 95% CI [0.03, 0.18]). Thus, Hypothesis 4b was proven, but not Hypothesis 3b.

Despite the apparent positive outcomes of VEGB, the third parties’ perceptions of VEGB are unclear. Is VEGB viewed positively or negatively by coworkers, and what are the behavioral outcomes of those evaluations? Existing work has shown that employees can react very differently to experiencing VEGB. The purpose of this manuscript was to identify factors that elicit different responses, and examine the potential for evaluations through social perception, and ultimately coworkers’ behavioral reactions to VEGB. The results suggest that VEGB can be perceived as both competence and warmth and that the nature of this evaluation may be dependent upon the attributions that coworkers make about employee motives for VEGB. Moreover, the perception that emerges from VEGB elicits different reactions from coworkers by engaging in green advocacy. Specifically, the results of our study indicate that observed VEGB indirectly influences the social perception and behavioral responses of coworkers at different levels of instrumental and moral attribution. When coworkers attributed VEGB to high levels of instrumental motives, observing VEGB evoked less competence and warmth perception. When coworkers attributed VEGB as having a high level of moral motive, witnessing VEGB elicited more competence and warmth perception. The social perception experienced by the employees motivated specific action tendencies, such as green advocacy.

RETRACTED

## Conclusion, implications, and future prospects

The VEGB appears to be good for the company, and it is equally important to understand whether VEGB is good for colleagues as well. As research on VEGB flourishes, there is a growing need for a comprehensive framework that explains why, how, and when coworkers respond differently to VEGB. We present a theoretical framework to explain the distinct social perception mechanisms and attribution constraints that would make it possible for VEGB to have fewer positive or negative effects on the conduct of coworkers. In particular, we have shown empirically that perceptions of warmth and competence mediated the relationship between VEGB and green advocacy, with differing motive attributions as a constraint.

### Theoretical implications

This investigation contributes to the VEGB and green advocacy literature in three ways. First, we integrate attributions and social perception perspectives to explain the complexity of coworkers’ responses to VEGB. We introduce the idea that motive attributions determine whether VEGB responds with warmth and competent cognition and the associated behaviors. The uncertainty of the attributed motions behind VEGB was considered a crucial aspect of the set by academics.

Second, we suggest that the psychological mechanisms underpinning VEGB’s influence on green advocacy include perceived competence and warmth. In the VEGB context, perceived warmth and competence are essential because such judgments are strongly related to coworkers’ perceptions of how skillful and caring employees are (Stauss, 2002). However, the notion of warmth and competence has received little attention in VEGB research. These results provide a complete picture and fill a research gap regarding the theories and mediating processes explaining why VEGB is linked to coworker outcomes.

Third, we explored the outcomes of VEGB in the workplace. Although previous studies have examined how context and individual characteristics affect VEGB (Norton et al., 2015; Kim et al., 2017), much attention has been focused on how VEGB helps organizations achieve environmental sustainability. Notably, it is yet unknown how VEGB works to elicit the attitudes and behaviors of coworkers. Thus, we try to fill this significant research gap regarding coworkers’ attribution by investigating how VEGB affects coworker green behaviors.

### Practical implications

Our study provides crucial information for managers and companies that are operating VEGB programs. Organizations are under increasing pressure to achieve their environmental goals. This study shows that coworkers’ perceptions of VEGB reciprocate the organizations by invoking green advocacy. The importance of organizations regularly informing their staff on VEGB programs, events, and environmental policies cannot be overstated. The organizations can organize meetings and workshops to raise awareness of VEGB activities. Therefore, organizations may benefit from embracing VEGB practices if they want to promote more pro-environmental involvement and behaviors within their workforce.

RETRACTED

Moreover, we point to the importance of coworkers’ attribution in these opinions. Coworkers are likely to have different perspectives on certain activities. For instance, our findings demonstrate that views on VEGB can range greatly, from favorable to unfavorable. Usually, employees are not well informed about VEGB. Managers who pay little attention to the impact of VEGB on coworkers may face unexpected organizational consequences in the form of less green advocacy. Sometimes employees honestly try to progress society and the environment, but coworkers perceive VEGB activities with attribution bias and doubt due to lack of communication. Managers should also address coworkers’ worries and skepticism about social responsibility activities by communicating clearly and frequently about VEGB actions using media such as WeChat, formal reports, seminars, and training programs. In this regard, VEGB must be genuine and not manipulative if it is to foster widespread employee perceptions of caring for the betterment of the environment.

### Limitations and future prospects

Some limitations could be resolved in further research. First, there is a possibility that correlations will be overstated and causality may be in doubt because coworkers reported the variables in our field study. Given that coworkers’ perceptions and attributions are most valid by self-report, we collected data from the same source at two time points to examine the relationship. However, the cross-sectional research design limits the validity of causality. Therefore, future research should use longitudinal designs or studies to examine coworkers’ reactions to VEGB.

Second, although we considered two attributed motives for VEGB, moral and instrumental concern, we did not examine the possible interaction between these motives. Future studies on VEGB motives could explore how they coexist or perhaps conflict with one another. Moreover, coworkers may be influenced by other aspects of individual differences and factors, beyond their motives, such as actors’ performance.

Third, future research should take into account other coworkers’ behavioral reactions. For example, coworkers may try to encourage employees to engage in more supportive or exclusive behaviors toward the actor. Moreover, they may have different opinions about the specific type of green behavior, such as required employee green behavior.

RETRACTED

## Data availability statement

The raw data supporting the conclusions of this article will be made available by the authors, without undue reservation.

## Ethics statement

Ethical review and approval was not required for the study on human participants in accordance with the local legislation and institutional requirements. Written informed consent for participation was not required for this study in accordance with the national legislation and the institutional requirements.

## Author contributions

XZ contributed to the conceptualization, data curation, and original draft preparation. ZL contributed to the supervision, methodology, reviewing, and editing. HZ contributed to the software, analysis, reviewing, and editing. QZ contributed to the resources, project administration, and funding acquisition. All authors contributed to the article and approved the submitted version.
